RETRACTED

# Study of Trunk Morphological Imbalance and Rehabilitation Outcome of Adolescent Idiopathic Scoliosis with Intelligent Medicine

**DOI:** 10.1155/2022/6775674

**Published:** 2022-03-29

**Authors:** Qin Zhao, Yiming Huang, Maodong Wu, Longying Shen, Yu Lu, Xingyue Fan, Qinglun Su

**Affiliations:** ^1^The First affiliated Hospital of Kangda College of Nanjing Medical University, Lianyungang, Jiangsu 222000, China; ^2^Department of Rehabilitation Medicine The First People's Hospital of Lianyungang, Lianyungang,, Liaoning 222000, China; ^3^Jinzhou Medical University Rehabilitation Medicine and Physiotherapy, Jinzhou 121001, Liaoning, China

## Abstract

In recent years, artificial intelligence technology has been widely used in various medical fields to effectively assist physicians in patient treatment operations. In this paper, we design and implement a deep biblical network model-based orthotic design for adolescent idiopathic scoliosis to quickly and effectively assist physicians in designing orthotics for adolescent idiopathic scoliosis. A fuzzy set is used to express the knowledge of adolescent idiopathic scoliosis orthosis design, and a fuzzy reasoning based on the confidence level is implemented. Finally, the efficiency of the design of adolescent idiopathic scoliosis orthoses was improved by 50% through two cases of adolescent idiopathic scoliosis patients, and the deviation rate between the inference value and the actual operation value of the domain experts was less than 10%.

## 1. Introduction

Adolescent Idiopathic Scoliosis (AIS) is a skeletal and muscular disorder of unknown etiology that occurs during preadolescence or before skeletal growth and maturation, mostly in females aged 10 to 18 years. The prevalence of scoliosis in adolescents is increasing year by year, and the prevalence of scoliosis in adolescents is reported to be more than 5% in Guangdong and other regions [1–3], and the increase in prevalence is especially obvious in junior high school (12–15 years old).

AIS can cause great physical and psychological harm to the affected adolescents and one of the most easily detected and most important concerns of the patients themselves is the physical appearance deformity. The most easily recognized and most important concern is the deformity of the physical appearance. Since the human torso is an integral part [4], AIS not only manifests as distortion and deformity of the spine but also affects the position of the scapular girdle, thorax, and pelvis, resulting in high and low shoulders, razor backs, thoracic deformities, and pelvic disorders [5, 6].

If left untreated, it can lead to secondary symptoms such as chronic pain and pulmonary dysfunction, and severe scoliosis deformity can also can cause irreversible damage to respiratory function and spinal nerves, bringing great harm to individuals and families [5]. Therefore, the prevention and treatment of the prevention and treatment of AIS has been the focus of attention of experts and scholars in the field of spinal surgery and spinal rehabilitation for patients with idiopathic scoliosis and their corresponding X-ray images, as shown in Figure 1.

RETRACTED

Surgery is recognized as an effective treatment for AIS, but according to statistics, only 1% of AIS patients require surgery and surgery can cause limitations in spinal motion. In Europe, exercise therapy interventions for scoliosis were first developed and have resulted in many mature rehabilitation systems; in China, research on AIS rehabilitation started later and there are more case studies and interventions [7, 8]. Therefore, experimental research on the idea or system of AIS rehabilitation therapy is needed.

Since the Cobb angle became the gold standard for scoliosis, the focus of AIS treatment has been on how to reduce the scoliosis angle and slow the progression of the scoliosis curve, while the local or overall morphological imbalance of the trunk caused by scoliosis has been increasingly neglected. Because the visual impact of poor posture is more severe, it is important to assess the trunk imbalance in patients with AIS before developing a rehabilitation program and to design a customized program for the patient [9].

AIS, as shown in Figure 2, is one of the most common types of scoliosis, accounting for approximately 80% of all idiopathic scoliosis, with the prevalence of AIS reaching 1% to 3% in the 10- to 16-year-old risk group. AIS not only affects the physical appearance of adolescents but also impairs their respiratory function, motor function, psychological status, and overall quality of life [10].

It is proposed that the difference of about 5° in scoliosis measurements is usually an error in measurement rather than a difference in the degree of scoliosis itself.

AIS is a common orthopedic disorder of uncertain etiology that affects the normal growth and function of the spine. 1%–3% of the normal population has AIS, and the main principle of clinical intervention is to control the progression of scoliosis using AIS orthoses [11–13]. An expert system contains a large amount of knowledge of domain experts inside and it can simulate the expert's reasoning methods to solve problems in the domain [14–16]. The currently popular expert systems are mainly classified as rule-based reasoning-based expert systems [17–20], artificial neural network-based expert systems [21], and rough set-based expert systems [22]. In [23], a generative-based expert system shell design method was proposed and applied to the treatment of AIS; however, the system could not be fully applicable to the knowledge expression and reasoning of uncertain information in the design of AIS orthoses.

RETRACTED

## 2. Related Work

The authors of [24] found that the Cobb angle measurement error was around 3.2°, and this measurement difference should be taken into account when diagnosing and treating scoliosis. In addition, errors in the Cobb angle measurement can lead to differences in subsequent staging. The typing reliability of radiographs based on a given angle was found by [24]. The authors of [25], only general intraobserver (*κ* = 0.50) and interobserver reliability (*κ* = 0.60) were found for Lenke typing in cases where the ab initio Cobb angle measurements were required. The authors of [2] proposed that T1 tilt signifies that patients may have upper thoracic segment scoliosis and validated that this method of determining the presence or absence of upper thoracic curvature was included in the King typing, but subsequent studies by [3] reported that patients with AIS with T1 tilt do not necessarily show differences in the appearance of high and low shoulders, and therefore, the T1 tilt direction and T1 tilt angle do not reflect the imbalance of the patient's shoulders. In [14], the angle between the line connecting the highest points of the left and right clavicles and the horizontal plane was defined as the clavicle angle (CA) and used as a parameter to measure the balance of the shoulder. A study by [7] showed a significant correlation between reduced cervical physiological curvature and inadequate thoracic kyphosis in patients with AIS; in addition, cervical curvature correlated with lumbar anterior convexity angle, independent of thoracolumbar lateral bending angle and pelvic parameters. Reference [6] performed an imaging study of sagittal pelvic parameters in normal Chinese adults and concluded that the mean value of PI in Chinese adults was 45.1° ± 9.6°.

In the field of spinal surgery, AI is widely used for diagnosis of diseases, especially for image processing, measurement, and classification. Theoretically, the successful development and application of AI-based automated measurement systems will provide an objective, accurate, and rapid solution to these problems and improve the diagnosis and treatment of AIS patients.

## 3. U-Net-Based Scoliosis Typing Algorithms for Idiopathic Scoliosis

The original data set is expanded, and the expanded data set is fed into the network for training and prediction to obtain the segmentation results; then, the segmentation results are fed into the automatic Cobb angle measurement algorithm designed in this paper to obtain the identified upper and lower endplate positions and Cobb angles; finally, the center points of the segmented images are extracted and fitted to obtain the curve fitting coefficient features, and the corresponding Cobb angles are measured by the automatic Cobb angle measurement algorithm. Finally, the center point of the segmented image is extracted and fitted to obtain the curve fitting coefficient features, and the corresponding bending bits and Cobb angles of the side slices are measured by the automatic Cobb angle measurement algorithm and used as auxiliary feature materials. The overall framework is shown in Figure 3, and the automatic Lenke typing algorithm based on the U-net partition network can be implemented by experimenting according to the process shown in the overall framework.

RETRACTED

## 4. Overall Design

The AIS expert system infers diagnostic and therapeutic solutions to assist physicians in solving complex medical problems [19]. The method in this paper can reason out the selection and design parameters of the AIS orthosis from patient information, and its structure is shown in Figure 4.

The architecture functional modules in this paper include the fuzzy reasoner, knowledge base, knowledge base management system, agenda, interpreter, and human-machine interface. They are described separately as follows. They activate rules from the knowledge base for questions posed by the user according to the established reasoning strategy and process the facts until the end of reasoning. A dynamic storage space containing all facts in the fact base and intermediate results in the reasoning process is present.

Real-time operations such as adding, deleting, modifying, and querying the knowledge base, as well as consistency and integrity checking of the knowledge therein are performed.

A database for storing domain expert knowledge is found. The knowledge base serves as the basis for reasoning and is the foundation of the expert system's reasoning.

A functional module explains the reasoning process of an expert system in a way that is easy to understand by the user. It gives the user a clear understanding of the reasoning process and decision making of the expert system.

The functional module that performs real-time operations such as adding, deleting, modifying, and querying the fact database, as well as displaying the expert system decisions and explanations by the interpreter is present.

The workflow of the method in this paper is shown in Figure 5.

Its fuzzy reasoning unit is shown in Figure 6.

In the fuzzy inference stage of the method in this paper, the confidence degree CFRHS of the right-hand side (RHS) of the activation rule is calculated as [10].

(1) $$\begin{array}{c} CF_{RHS}=CF_{LHS}\times CF_{R}, \end{array}$$

where CFLHS is the confidence of the left part of the rule; CR is the confidence of the rule.

RETRACTED

In the deblurring stage, the deblurring algorithm of the method in this paper uses the weighted average method [21], which is given as follows:

(2) $$\begin{array}{c} x=\frac{\sum_{i=1}^{n}x_{i}\mu \left(x_{i}\right)}{\sum_{i=1}^{n}\mu \left(x_{i}\right)},\left(n=1,2,3,\cdots \right), \end{array}$$

where *x* is the clear amount of design parameters; *x*_*i*_ is the value of fuzzy subset; *μ*(*x*_*i*_) is the affiliation degree of fuzzy subset.

The AIS orthosis is then shaped and manufactured from the patient's phantom according to the shaping volume. After the patient has tried on the AIS orthosis, the doctor determines the amount of trim adjustment for the AIS orthosis based on the patient's feedback and adjusts the trim of the AIS orthosis according to the amount of trim adjustment. By adjusting the height of the pressure application zone of the AIS orthosis, the orthotic force exerted on the patient is thereby adjusted until the patient no longer experiences discomfort while wearing the orthosis [23]. As shown in Figure 7, the determination of the amount of trim and trim adjustment is an important factor in ensuring that the AIS orthosis meets the individual needs of the patient.

The fact sheet in the knowledge base management system is used to maintain the known facts in the fact base. The knowledge engineer conceptualized and formalized 848 AIS treatment and AIS orthotic design rules through interviews and case studies with AIS conservative treatment specialists [26].

## 5. Application Examples

To verify the feasibility of the proposed expert system design method for AIS orthosis design based on the fuzzy reasoning, the method in this paper was applied to the AIS orthosis-assisted design of 2 cases of AIS patients.

The method in this paper was successfully applied to the AIS orthosis-assisted design of 2 AIS patients. The average design time of the AIS orthoses for Patient A and Patient B was reduced from 4 h to 2 h with the aid of this method, which improved the design efficiency of the AIS orthoses by 50% as shown in Figure 8. The deviation rates of some of the methods in this paper are shown in Table 1, and the deviation rates of the inferred values from the actual operational values of the domain experts in the AIS orthosis design of this paper are less than 10%. This shows that the method of this paper can assist physicians in designing AIS orthoses quickly and efficiently.

RETRACTED

## 6. Experimental Analysis

The raw data of the spine were provided by Shenzhen University General Hospital, and the spine segmentation performed in this chapter The experiments were performed for the thoracic, lumbar, and full spine segmentation of the orthopantomographs of the spine. Among them, the original data volume of lumbar spine was 84. The original data volume for the lumbar spine was 84 cases, the original data volume for the thoracic spine was 166 cases, and the original data volume for the coronal position was 88 cases. Each of these cases is derived from different patient x-rays. Since the original data could not be trained for deep learning, the data were expanded by rotation, flip, and offset [27, 28]. The expanded data were 1050 for lumbar spine, 4910 for thoracic spine, and 6302 for coronal spine. The size of the data expansion was determined by the ease of segmentation. The experimental platform is based on the Window 7 system and the Kares deep learning library.

From the training process, in Figure 9, the Loss curves of the training and validation sets show a steady decreasing trend, and the IOU shows an increasing trend overall. After 50 iterations, the loss values of the training and validation sets of the lumbar spine drop to 0.033 and 0.0754, and the loss values of the training and validation sets of the thoracic spine drop to 0.0537 and 0.050. The IOU values of the training and validation sets of the thoracic spine can reach 0.6341 and 0.6342, and the IOU values of the training and validation sets of the lumbar spine can reach The training and validation sets for the lumbar spine were 0.5947 and 0.5948, respectively.

The training process of full spine segmentation is shown in Figure 10 below, from which we can see that the red discounted represents the improved U-net model and the blue-dashed line represents the original U-net model. The improved U-net model is able to segment the contours of the coronal spine well, and it is very meaningful for medical diagnosis to be able to achieve the segmentation of the coronal position. With good segmentation results, the accuracy of the subsequent series of automatic measurements will also be improved.

## 7. Conclusions

The accuracy rate of the system in this paper is more than 80%. The above studies are all applications of the expert system technology in the direction of scoliosis-assisted diagnosis and treatment and have achieved a certain accuracy rate, but their inference models have not yet reached the optimal accuracy rate. The main reason for this is the use of the traditional generative reasoning model, which relies on the physician's empirical knowledge in the treatment of scoliosis and contains a large amount of uncertain information. Fuzzy logic is a method that can effectively handle uncertain information based on multivalued logic and can effectively realize the expression and inference of uncertain knowledge in expert systems. The future research direction should be to further investigate the influence of individual and gender differences on this method by increasing the number of subjects.

RETRACTED

## Figures and Tables

**Figure 1:** Patients with idiopathic scoliosis and their corresponding x-ray images.

**Figure 2:** Cobb angle measurement method.

**Figure 3:** Flowchart of the overall framework of the U-net-based automatic typing algorithm.

**Figure 4:** Structure of the scoliosis orthosis design expert system (SODES).

**Figure 5:** Workflow diagram of the expert system.

**Figure 6:** Fuzzy inference unit of the scoliosis orthosis design expert system.

**Figure 7:** “Three point force” orthopedic diagram.

**Figure 8:** Patients A and B wearing the scoliosis orthosis design expert system (method in this paper) assisted by the before and after comparison of adolescent idiopathic scoliosis orthoses designed with the aid of the design expert system.

**Figure 9:** Data display of the thoracolumbar spine training process.

**Figure 10:** Training results of the U-net network and its improved network in coronal position.

**Table 1:** Deviation rate of the expert system component.

Project	Patient A				Patient B			
	Opening diameter of release area (CM)	Opening angle of release area (°)	Three-point force modification (CM)	Adjustment amount of three-point force repair (CM)	Opening diameter of release area (CM)	Opening angle of release area (°)	Three-point force modification (CM)	Adjustment amount of three-point force repair (CM)
Inference value	15.8	54.8	6.3	1.5	14.5	48.4	5.1	2
Recommended value	15	60	6	1.6	14.9	52	5.5	1.8
Deviation rate	5%	9.4	4.7	6.7	3.4	7.4	7.8	10

## Data Availability

The data underlying the results presented in the study are available within the manuscript.
